# Hypochlorous acid via peroxynitrite activates protein kinase Cθ and insulin resistance in adipocytes

This article has been retracted.

**DOI:** 10.1530/JME-14-0213

**Published:** 2015-02

**Authors:** Jun Zhou, Qilong Wang, Ye Ding, Ming-Hui Zou

**Affiliations:** 1 Section of Molecular Medicine, BSEB 306A, Department of Internal Medicine, University of Oklahoma Health Sciences Center, Oklahoma City, Oklahoma, 73104, USA

**Keywords:** hypochlorous acid, insulin resistance, IRS1, peroxynitrite

## Abstract

We recently reported that genetic deletion of myeloperoxidase (MPO) alleviates obesity-related insulin resistance in mice *in vivo*. How MPO impairs insulin sensitivity in adipocytes is poorly characterized. As hypochlorous acid (HOCl) is a principal oxidant product generated by MPO, we evaluated the effects of HOCl on insulin signaling in adipocytes differentiated from 3T3-L1 cells. Exposure of 3T3-L1 adipocytes to exogenous HOCl (200 μmol/l) attenuated insulin-stimulated 2-deoxyglucose uptake, GLUT4 translocation, and insulin signals, including tyrosine phosphorylation of insulin receptor substrate 1 (IRS1) and phosphorylation of Akt. Furthermore, treatment with HOCl induced phosphorylation of IRS1 at serine 307, inhibitor κB kinase (IKK), c-Jun NH_2_-terminal kinase (JNK), and phosphorylation of PKCθ (PKCθ). In addition, genetic and pharmacological inhibition of IKK and JNK abolished serine phosphorylation of IRS1 and impairment of insulin signaling by HOCl. Furthermore, knockdown of PKCθ using siRNA transfection suppressed phosphorylation of IKK and JNK and consequently attenuated the HOCl-impaired insulin signaling pathway. Moreover, activation of PKCθ by peroxynitrite was accompanied by increased phosphorylation of IKK, JNK, and IRS1-serine 307. In contrast, ONOO^−^ inhibitors abolished HOCl-induced phosphorylation of PKCθ, IKK, JNK, and IRS1-serine 307, as well as insulin resistance. Finally, high-fat diet (HFD)-induced insulin resistance was associated with enhanced phosphorylation of PKCθ, IKK, JNK, and IRS1 at serine 307 in white adipose tissues from WT mice, all of which were not found in *Mpo* knockout mice fed HFDs. We conclude that HOCl impairs insulin signaling pathway by increasing ONOO^−^ mediated phosphorylation of PKCθ, resulting in phosphorylation of IKK/JNK and consequent serine phosphorylation of IRS1 in adipocytes.

## Introduction

Insulin resistance, a hallmark of obesity and fundamental cause of type 2 diabetes, is characterized by a diminished ability of insulin to regulate glucose homeostasis in insulin-sensitive organs including liver, skeletal muscle, and adipose tissue. Insulin resistance is partly caused by chronic low-level inflammation and oxidative stress in adipose tissue (Guo 2014). Infiltration of inflammatory cells, which produce cytokines and oxidants, leads to a local inflammatory environment in adipose tissue (Olefsky & Glass 2010). Accumulated evidence indicates that increased infiltration of neutrophils in adipose tissue is strongly related to the development of insulin resistance in human obesity (Elgazar-Carmon *et al*. 2008, Talukdar *et al*. 2012). Recently, we reported that neutrophil-derived myeloperoxidase (MPO) activation plays an important role in obesity-induced insulin resistance (Wang *et al*. 2014). Hypochlorous acid (HOCl) is a potent oxidant formed from hydrogen peroxide and chloride ions in a reaction catalyzed by MPO (Harrison & Schultz 1976). Recently, a high correlation between the production of HOCl and metabolic disorder was identified, i.e. the concentration of HOCl in plasma was elevated in obese subjects and hypertensive patients (Yang *et al*. 2013). In addition, HOCl-modified proteins were present in liver and adipose tissue of obese patients (Rensen *et al*. 2009). However, the molecular mechanism and role of HOCl in the pathogenesis of insulin resistance remain to be determined.

The insulin signaling transduction cascade initiated by insulin binding to its receptor causing receptor autophosphorylation and tyrosine phosphorylation of insulin receptor substrate 1 (IRS1) subsequently activating phosphoinositide 3-kinase and Akt and finally inducing translocation of intracellular GLUT4 vesicles to the cell membrane in order to enhance the uptake of glucose (Bevan 2001). Insulin resistance is caused by impaired insulin signal transduction accompanied by decreased activation of downstream obligate molecular intermediates (Saltiel & Kahn 2001). Accumulating lines of evidence have indicated that serine phosphorylation of IRS1 led to inhibition of insulin signals via interference with tyrosine phosphorylation of IRS1 and acceleration of its degradation (Gual *et al*. 2005). Moreover, activation of several inflammatory kinases, including inhibitor κB kinase (IKK), c-Jun NH2-terminal kinase (JNK), and protein kinase C (PKC), induces serine phosphorylation of IRS1 by inflammatory cytokines and pro-oxidants (Aguirre *et al*. 2000, Morino *et al*. 2005, Weigert *et al*. 2008). HOCl is known as a potent oxidant and a major inflammatory mediator inducing tissue injury in a number of inflammatory diseases (Souza *et al*. 2011). Therefore, we propose the hypothesis that HOCl mediates insulin resistance through activation of PKC, IKK, and JNK, resulting in subsequent serine phosphorylation of IRS1 in adipocytes. Here, we report that exogenous HOCl impaired the insulin signaling pathway and induced phosphorylation of IRS1 at Ser307, IKK, JNK, and PKCθ in 3T3-L1 adipocytes. In contrast, HOCl-impaired insulin signals were abolished after knockdown of IKKβ and JNK using siRNA or a pharmaceutical inhibitor. Moreover, PKCθ knockdown attenuated phosphorylation of IKK and JNK, resulting in restoration of insulin sensitivity. Strikingly, exogenous HOCl-induced insulin resistance and phosphorylation of PKCθ were prevented by an ONOO^−^ scavenger. Overall, our findings provide a novel mechanistic basis for understanding how MPO-derived HOCl mediates insulin resistance in adipocytes.

## Materials and methods

### Materials

Mouse 3T3-L1 preadipocytes were obtained from American Type Culture Collection (Manassas, VA, USA). 3T3-L1 preadipocyte medium, 3T3-L1 adipocyte differentiation medium, and 3T3-L1 adipocyte maintenance medium were obtained from Zen-Bio, Inc. (Research Triangle Park, NC, USA). [1,2-^3^H] 2-deoxy-d-glucose was purchased from Perkin Elmer Life Sciences (Waltham, MA, USA). Hypochlorous sodium solution, human insulin, *N*ω-nitro-l-arginine methyl ester hydrochloride (l-NAME), SP600125, and antibody against phospho-IRS1 (Tyr612) were purchased from Sigma–Aldrich. Protein A/G-agarose, RIPA lysis buffer, PS-1145, IKKβ siRNA, JNK2 siRNA, PKCθ siRNA, control siRNA, and antibodies against β-actin, GAPDH, and Na^+^/K^+^ ATPase were obtained from Santa Cruz Biotechnology, Inc. Antibodies against phospho-IRS1 (Ser307), IRS1, phospho-Akt (Ser473), phospho-Akt (Thr308), Akt, phospho-GSK3β (Ser9), GSK3β, phospho-IKKα/β (Ser176/180), IKKα, IKKβ, phospho-SAPK/JNK (Thr183/Tyr185), JNK, phospho-PKCθ (Thr538), PKCθ, GLUT4, IκBα, and HRP-linked secondary antibodies were purchased from Cell Signaling Technology (Beverly, MA, USA). ONOO^−^ was obtained from Calbiochem (Billerica, MA, USA). All other chemicals were of the highest commercial grade available.

### Cell treatment

3T3-L1 preadipocytes were cultured and differentiated into adipocytes as described previously (Worrall & Olefsky 2002). By days 8–12 after induction of differentiation, more than 90% of the cells exhibited the characteristic lipid-vesicle-filled adipocyte phenotype. After overnight incubation in DMEM supplemented with 0.1% BSA, 3T3-L1 adipocytes were exposed to various concentrations of HOCl in the presence of 0.1% BSA for 1 h. HOCl-treated 3T3-L1 adipocytes were further stimulated with insulin for 15 min. HOCl was prepared by treating hypochlorous sodium with hydrochloric acid to adjust the pH to 4.0 according to a protocol published previously (Wang *et al*. 2007). The concentrations of HOCl were determined spectrophotometrically at 292 nm in 0.1 mol/l NaOH (*ϵ*=350/(mol/l) per cm).

### 2-Deoxyglucose (2-DG) uptake

The glucose uptake was assayed as described previously (Worrall & Olefsky 2002). Following overnight serum starvation, adipocytes were starved of glucose for 1 h in HEPES buffer containing 0.1% BSA and exposed to different concentrations of HOCl for 1 h. Then, cells were stimulated with 100 nM insulin for 15 min following addition of 0.2 μCi [1,2-^3^H] 2-DG for 5 min. Finally, cells were washed three times with ice-cold PBS buffer and solubilized with 1% Triton X-100. ^3^H-2-DG uptake was determined using a liquid scintillation counter. The intracellular concentration of 2-DG was normalized to total protein content.

### Western blotting analysis

Proteins were extracted from 3T3-L1 cells with RIPA lysis buffer (Santa Cruz Biotechnologies) containing 1 mM Na_3_VO_4_, 1 μg/ml leupeptin, and 1 mM phenylmethylsulfonyl fluoride. Protein concentration was measured using the BCA method (Pierce, Rockford, IL, USA). Cell lysates were resolved by SDS–PAGE and transferred to PVDF membrane (Millipore Corp., Bedford, MA, USA). Membranes were blocked with 5% milk and probed with specific antibodies and subsequently incubated with HRP-linked secondary antibodies. Proteins were visualized using an ECL detection system (Pierce).

### siRNA transfection

IKKβ, JNK1, PKCθ, and control siRNA (10 μmol/l) were added to OPTI-MEM-reduced serum media (Life Technologies) with Lipofectamine RNAiMAX (Invitrogen Corp.). Adipocytes in six-well plates were transfected with siRNA in transfection medium for 6 h. The transfection medium was then replaced with a culture medium containing 10% FBS and incubated for 48 h.

### Assay of *in vitro* Akt kinase activity

A total of 500 μg protein was incubated with anti-Akt antibody and Sepharose beads overnight at 4 °C. After binding, the beads were washed four times with lysis buffer. Akt activity was measured using a non-radioactive Akt kinase assay kit (Cell Signaling Technology, Inc., Beverly, MA, USA).

### Experimental animals

MPO knockout (*Mpo* ^−^^*/*^^−^) mice were purchased from The Jackson Laboratory (Bar Harbor, ME, USA). C57BL/6J mice were used as WT controls. Mice were housed in temperature-controlled cages under a 12 h light:12 h darkness cycle. Starting at 6 weeks of age, male mice were fed a high-fat diet (HFD, D12492; Research Diets, New Brunswick, NJ, USA) consisting of 60% fat, 20% protein, and 20% carbohydrate or a normal chow diet (ND) consisting of 13% fat, 29% protein, and 58% carbohydrates (LabDiet, St Louis, MO, USA) for up to 16 weeks. At the end of the experiments, mice were fasted for 6 h. Body weight and food intake were measured. Blood samples were collected for detecting fasting glucose and plasma insulin (ALPCO, Salem, NH, USA). Epididymal white adipose tissue (WAT) was collected and stored at −80 °C. The animal protocol was reviewed and approved by the University of Oklahoma Institutional Animal Care and Use Committee.

### Immunohistochemical analysis

Epididymal WAT from HFD-fed WT and *Mpo* ^−^^*/*^^−^ mice were fixed in 4% paraformaldehyde for 16 h and embedded in paraffin. Sections were deparaffinized, rehydrated, and microwaved in citrate buffer for antigen retrieval. Sections were successively incubated in 3% hydrogen peroxide, protein block buffer, and primary antibody against HOCl-oxidized LDL (Millipore Corp.) antibody against 3-chlorotyrosine (Hycult Biotech. PA, USA) overnight at 4 °C. Then, sections were rinsed in PBS buffer and incubated with labeled polymer-HRP anti-rabbit antibody and DAB chromogen.

### Statistical analysis

Values are expressed as mean±s.e.m. One-way ANOVA was used to compare the differences among the three groups followed by Bonferroni's multiple comparison tests as applicable, and *P*<0.05 was considered significant.

## Results

### HOCl impairs insulin-stimulated glucose uptake, insulin signals, and GLUT4 translocation

We first investigated the effect of HOCl on insulin-stimulated glucose uptake measurement with 2-deoxyglucose (2-DG) labeled with tritium in 3T3-L1 adipocytes. Results of previous studies by our group and other laboratories (Ginion *et al*. 2011, Liu *et al*. 2013) on time–action and dose–response curves for insulin-stimulated glucose uptake revealed that stimulation with 100 nmol/l insulin for 15 min could induce maximal insulin action, this dose was used for the entire study to induce glucose uptake and transduction of transduction of insulin signaling in 3T3-L1 adipocytes. HOCl dose-dependently decreased insulin-stimulated glucose uptake but not the basal rate of glucose uptake, indicating an insulin-resistant state. Treatment with HOCl at a pathologically relevant oxidant concentration (200 μmol/l; Hawkins *et al*. 2001) resulted in approximately 70% suppression of uptake of glucose (Fig. 1A). Therefore, 200 μmol/l HOCl was used to treat adipocytes in the subsequent experiments. Insulin could induce translocation of GLUT4 to the cellular membrane, which increases the uptake of glucose into the cells. Treatment with HOCl inhibited insulin-stimulated translocation of GLUT4 to the plasma membrane, while not affecting the expression of GLUT4 in the whole-cell lysates (Fig. 1B).

Next, we measured the molecular targets of HOCl-induced changes in glucose uptake. Insulin treatment stimulated phosphorylation of IRS1 at Tyr612 (Fig. 2A), Akt, and its downstream substrate GSK3β. Pretreatment of adipocytes with HOCl inhibited insulin-induced phosphorylation of Akt and GSK3β (Fig. 1C). In parallel, treatment with HOCl suppressed the activity of Akt kinase as evaluated by phosphorylation of GSK3β fusion protein (Fig. 1D). These results indicated that treatment with HOCl induced insulin resistance in adipocytes.

### HOCl promotes phosphorylation of IRS1 at Ser307, IKK, and JNK

Results from recent studies indicated that serine phosphorylation of IRS1, mediated by JNK and IKK, was associated with inhibition of the insulin signaling pathway by inflammatory cytokines (Aguirre *et al*. 2000, Morino *et al*. 2005, Weigert *et al*. 2008). Thus, we examined the effect of HOCl on serine phosphorylation of IRS1 at residue 307. As shown in Fig. 2A, HOCl treatment dramatically increased phosphorylation of IRS1 at Ser307 in the presence or absence of insulin, but not the expression of IRS1. Meanwhile, insulin-stimulated tyrosine phosphorylation of IRS1 was suppressed after pretreatment with HOCl. In parallel, treatment with HOCl dramatically increased phosphorylation of IKKα/β at Ser176/180 and JNK at Thr183/Tyr185, but not protein expression (Fig. 2B and C).

### Phosphorylation of IKKβ is involved in HOCl-induced insulin resistance

Next, we investigated whether IKKα/β was required for HOCl-triggered phosphorylation of IRS1-Ser307 and insulin resistance. To this end, the IKK-selective inhibitor PS-1145 (10 μmol/l) was used to pretreat adipocytes before the addition of HOCl. PS-1145 suppressed HOCl-induced phosphorylation of IKKα/β and reduced serine phosphorylation of IRS1 at 307. Furthermore, PS-1145 significantly abrogated HOCl-impaired insulin signals, including tyrosine phosphorylation of IRS1 and phosphorylation of Akt and GSK3β (Fig. 3A). To confirm this result, IKKβ-specific siRNA was used to suppress the expression of IKK and then HOCl-impaired insulin signals were evaluated. IKKβ siRNA significantly decreased the expression of IKKβ and HOCl-induced phosphorylation of IKKβ. Furthermore, IKKβ siRNA attenuated serine phosphorylation of IRS1 at position 307 and restored phosphorylation of IRS1 at Tyr612, phosphorylation of Akt and GSK3β by insulin (Fig. 3B). These data provide strong evidence that IKKβ is required for serine phosphorylation of IRS1 at position 307 and impairment of insulin signaling after treatment with HOCl.

### Phosphorylation of JNK is required for HOCl-induced insulin resistance

We also determined whether phosphorylation of JNK mediated phosphorylation of IRS1-Ser307 and insulin resistance after stimulation with HOCl. As expected, the JNK-specific inhibitor SP-600125 (30 μmol/l) markedly suppressed HOCl-induced phosphorylation of JNK phosphorylation accompanied by serine phosphorylation of IRS1 at 307 residues. In parallel, SP-600125 significantly abrogated the HOCl-induced impairment of insulin signals, as demonstrated by the restoration of phosphorylation of IRS1 at Tyr612, Akt, and GSK3β by insulin (Fig. 4A).

Next, we assayed whether genetic suppression of JNK altered the HOCl-impaired insulin signaling pathway. As shown in Fig. 4B, transfection with JNK siRNA significantly decreased the expression and HOCl-induced phosphorylation of JNK. Also HOCl-induced phosphorylation of IRS1 at Ser307 was dramatically decreased in cells transfected with JNK, compared with control. Moreover, JNK siRNA abrogated HOCl-impaired insulin signaling, as demonstrated by restoration of insulin-stimulated tyrosine phosphorylation of IRS1 and phosphorylation of Akt and GSK3β. These results indicate that phosphorylation of JNK is required for insulin resistance and phosphorylation of IRS1 at Ser307 in 3T3-L1 adipocytes treatment with HOCl.

### PKCθ mediates HOCl-induced insulin resistance via activation of IKK and JNK

PKCθ could activate IKKβ and JNK, leading to phosphorylation of IRS1 at Ser307 and Ser302 (Werner *et al*. 2004). Thus, we verified whether activation of PKCθ contributes to HOCl-induced phosphorylation of IKK and JNK and insulin resistance. Exposure of 3T3-L1 adipocytes to HOCl induces phosphorylation of PKCθ at Thr538. Also knockdown of PKCθ by siRNA transfection partly attenuated HOCl-induced phosphorylation of IKK and JNK, indicating that HOCl activates IKK and JNK in a PKCθ-dependent manner (Fig. 5A). In parallel, transfection with PKCθ siRNA dramatically decreased HOCl-induced serine phosphorylation of IRS1 at residue 307 and restored insulin-stimulated tyrosine phosphorylation of IRS1 (Fig. 5B). Moreover, PKCθ siRNA partially recovered insulin-enhanced Akt kinase activity (Fig. 5C) and translocation of GLUT4 to the plasma membrane (Fig. 5D). Taken together, these results indicate that PKCθ phosphorylation is involved in HOCl-induced insulin resistance via activation of IKK and JNK in 3T3-L1 adipocytes.

### ONOO^−^ mediates phosphorylation of PKCθ and IRS1-Ser307 after HOCl treatment

Our group has demonstrated that HOCl enhanced ONOO^−^ production, a potent oxidative molecular formed by superoxide (O_2_·^−^) and nitric oxide (NO) (Wang *et al*. 2014). Also ONOO^−^ plays a causal role in the pathogenesis of insulin resistance in obesity and type 2 diabetes (Randriamboavonjy & Fleming 2009). To determine whether ONOO^−^ was involved in HOCl-induced activation of inflammatory kinases and insulin resistance, 3T3-L1 adipocytes were preincubated with l-NAME (1 mmol/l) to inhibit the production of NO, Cu/Zn SOD (SOD1, 150 U/ml) to remove O_2_·^−^, or uric acid (50 μmol/l) to scavenge ONOO^−^ before stimulation with HOCl, and then phosphorylation of PKCθ, IKK, JNK, and IRS1 was evaluated. As shown in Fig. 6A, HOCl-induced phosphorylation of PKCθ was blocked by SOD1, l-NAME, and uric acid treatment. In addition, ONOO^−^ dose-dependently induced phosphorylation of PKCθ, but not expression of the protein (Fig. 6B), indicating that ONOO^−^ contributes to the phosphorylation of PKCθ by HOCl.

We further confirmed the role of ONOO^−^ in PKCθ-mediated downstream signals, including serine phosphorylation of IKK, JNK, and IRS1. As shown in Fig. 6C, SOD1, l-NAME, and uric acid suppressed phosphorylation of IKK, JNK, and IRS1-Ser307 in adipocytes treated with HOCl. In addition, ONOO^−^ dose-dependently induced phosphorylation of IKK and JNK. Meanwhile, ONOO^−^ increased serine phosphorylation of IRS1 and reduced tyrosine phosphorylation of IRS1 by insulin (Fig. 6D). Collectively, these results indicate that ONOO^−^ mediates HOCl-induced Ser307 phosphorylation of IRS1 via activation of PKCθ, IKK, and JNK.

### HOCl-induced insulin resistance is ONOO^−^ dependent

Pretreatment with SOD1, l-NAME, and uric acid prevented HOCl-induced impairment of insulin signals, as demonstrated by restoration of tyrosine phosphorylation of IRS1, phosphorylation of Akt, and Akt kinase activity by insulin (Fig. 7A, B and C). Moreover, SOD1, l-NAME, and uric acid abolished the deleterious effect of HOCl on translocation of GLUT4 to the plasma membrane (Fig. 7D). In contrast, the hydrogen peroxidase scavenger catalase offered no protection against HOCl-induced impairment of insulin signaling. Taken together, these results indicate that ONOO^−^ is involved in HOCl-induced insulin resistance.

### Deletion of MPO attenuates HFD-induced phosphorylation of IKK, JNK, and IRS1-Ser307

MPO is the sole mammalian oxidant enzyme to catalyze production of HOCl in the presence of hydrogen peroxide and chloride ions (Olza *et al*. 2012). To extend our *in vitro* findings, we measured the insulin signals and molecular pathway involved in insulin resistance in WT and MPO knockout (*Mpo* ^−^^*/*^^−^) mice. The initial body weights of WT and *Mpo* ^−^^*/*^^−^ male mice at 6 weeks of age were similar. After 16 weeks of HFD feeding, WT mice displayed higher body weights, fasting blood glucose, and plasma insulin levels than *Mpo* ^−^^*/*^^−^ mice. In parallel, high level of homeostasis model assessment of insulin resistance (HOMA-IR) indicated that WT mice developed severe insulin resistance than *Mpo* ^−^^*/*^^−^ mice (Table 1). In epididymal WAT of WT mice fed with HFD, infiltration of neutrophils (Wang *et al*. 2014), and expression of MPO were increased compared with ND-fed WT mice (Fig. 8A). In addition, 3-chlorotyrosine, a biomarker for HOCl, was present in the WAT from WT mice, mainly in the crown-like structure that contains neutrophils and macrophages. This 3-chlorotyrosine stain was absent in *Mpo* ^−^^*/*^^−^ mice (Fig. 8B). In parallel, HFD increased phosphorylation of IRS1 at Ser307, PKCθ, JNK, and IKK in WAT, while not affecting protein expression. However, the effect of HFD on phosphorylation of IRS1-Ser307, PKCθ, JNK, and IKK was absent in *Mpo* ^−^^*/*^^−^ mice (Fig. 8C and D).

## Discussion

This study has unveiled the mechanism whereby HOCl induces insulin resistance in adipocytes. We showed that a clinically relevant concentration of HOCl impairs insulin-stimulated glucose uptake, reduces the amplitude of the insulin signal, and enhances phosphorylation of IRS1 at serine 307. Most importantly, HOCl induces PKCθ-dependent activation of IKK/JNK by ONOO^−^, causing serine phosphorylation of IRS1 and insulin resistance (Fig. 8E).

The key lines of evidence can be summarized as follows: first, HOCl induces phosphorylation of IKK and JNK, whereas inhibition of IKK or JNK blocks serine phosphorylation of IRS1 and impairment of insulin signals. These results indicate that activation of both IKK and JNK by HOCl is required for insulin resistance; secondly, HOCl induces phosphorylation of PKCθ, and suppression of PKCθ attenuates phosphorylation of IKK/JNK and restores insulin-stimulated glucose uptake, implying that PKCθ serves as an upstream kinase of IKK/JNK; thirdly, ONOO^−^ treatment dose dependently induces phosphorylation of PKCθ, whereas an ONOO^−^ scavenger reduces HOCl-stimulated phosphorylation of PKCθ, IKK, JNK, and IRS1-Ser307. These results indicate that ONOO^−^ is the initial trigger for the development of insulin resistance in response to HOCl. Finally, deletion of MPO protects against HFD-induced phosphorylation of PKCθ, IKK, JNK, and IRS1-Ser307 accompanied by insulin resistance in WAT. Overall, our results indicate that ONOO^−^ mediated PKCθ-dependent serine phosphorylation of IRS1 might be responsible for HOCl-induced insulin resistance.

IRS1 is an essential insulin signal transducer for activating downstream signals after tyrosine phosphorylation. But serine/threonine phosphorylation of IRS1 exerts the opposite regulatory effect on insulin signaling via accelerated degradation and interference with tyrosine phosphorylation. Several inflammatory cytokines, such as tumor necrosis factor alpha (TNFα) and interleukin 1 beta (IL1β), induce serine phosphorylation of IRS1 at position 307 and insulin resistance. Interestingly, mutation of serine 307 to alanine (IRS1 S307A) causing dephosphorylation at this site eliminates TNFα-decreased tyrosine phosphorylation of IRS1 in Chinese hamster ovary cells, underlining the important inhibitory function of this site in transduction of insulin signaling (Aguirre *et al*. 2000). Weigert *et al*. (2008) confirmed that IRS1 S307A mutation enhanced phosphorylation of Akt in skeletal muscle cells. Consistently, muscle-specific mutations at IRS1-Ser302, 307, and 612 increased uptake of glucose and insulin signaling (Morino *et al*. 2008). Thus, we proposed the hypothesis that inhibition of tyrosine phosphorylation of IRS1 and impairment of the insulin signaling pathway might be due to serine phosphorylation of IRS1 by HOCl. Indeed, we found that treatment with HOCl increased serine phosphorylation of IRS1 at position 307 and reduced insulin-stimulated tyrosine phosphorylation of IRS1 in 3T3-L1 adipocytes. Interestingly, these opposite effects of HOCl on serine/tyrosine phosphorylation of IRS1 were simultaneously reversed after blockage of activation of serine/threonine protein kinases, including IKK, JNK, and PKCθ. These results are indicative of a significant negative association between serine phosphorylation at residue 307 and tyrosine phosphorylation of IRS1 in adipocytes. Consistent with the conclusion, serine phosphorylation of IRS1 also strongly correlates with impairment of the insulin signaling pathway in liver and muscle of diabetic mice and humans (Morino *et al*. 2005, Dong *et al*. 2008). Recently, this finding has been challenged by Copps and colleagues who global IRS1 S307A knock-in mice and observed insulin resistance in 5-month-old mice fed with a chow diet, indicating that IRS1-Ser307 makes a positive contribution to maintaining good insulin sensitivity (Copps *et al*. 2010). However, direct evidence is lacking to support the hypothesis that phosphorylation of IRS1-Ser307 causes inhibition of tyrosine phosphorylation and insulin resistance in adipocytes treated with HOCl. Further investigation is warranted.

The inflammatory kinases IKKβ and JNK serve as critical molecular links between obesity, metabolic inflammation, and insulin resistance. Activation of IKK and JNK could phosphorylate IRS1 on a number of serine residues, resulting in inhibition of insulin signaling. IL1β activates JNK1 and subsequently phosphorylates IRS1 at Ser307 in adipocyte (He *et al*. 2006). Another cytokine, TNFα, also IKK-dependently increases IRS1-Ser307 phosphorylation in 3T3-L1 adipocytes (Nakamori *et al*. 2006). Treatment with HOCl induces phosphorylation of JNK in primary biliary cells (Salunga *et al*. 2007) and activates NF-κB in endothelial cells (Pullar *et al*. 2002). Therefore, we propose the hypothesis that HOCl induces serine phosphorylation of IRS1 via activation of IKK and JNK. Indeed, exposure of 3T3-L1 adipocytes to HOCl significantly increases phosphorylation of JNK and IKK. In contrast, pharmaceutical inhibitors and siRNA-mediated knockdown of JNK and IKKβ prevent impairment of insulin signaling and phosphorylation of IRS1-Ser307, indicating that HOCl-mediated insulin resistance is dependent on activation of JNK and IKK. This conclusion is further supported by results from our *in vivo* studies indicating that knockout of MPO reduces phosphorylation of IKK, JNK, and IRS1-Ser307 in WAT, and in parallel protects against insulin resistance in HFD-fed obese mice.

PKCθ has been reported to induce phosphorylate of IRS1 on Ser307 and Ser302 via activation of IKKβ and JNK (Gao *et al*. 2004). Free fatty acid is an inducer of PKCθ phosphorylation, causing to cause development of insulin resistance in adipocytes (Gao *et al*. 2004) and skeletal muscle cells (Kadotani *et al*. 2009). In this study, we have demonstrated HOCl to be a novel mediator of activation of PKCθ in adipocytes, which might contribute to adipose inflammation and insulin resistance. Treatment with HOCl induced phosphorylation of PKCθ in 3T3-L1 adipocytes. Moreover, knockdown of PKCθ using siRNA transfection attenuated phosphorylation of IKK, JNK, and IRS1-Ser307 and restored impairment of the insulin signaling pathway by HOCl. These results indicate that PKCθ functions upstream of IKK and JNK to induce insulin resistance. It is noteworthy that knockdown of PKCθ could not fully inhibit HOCl-induced activation of IKK and JNK, indicating that treatment with HOCl may activate IKK and JNK in other ways independent of PKCθ. Besides PKCθ, PKCζ is also involved in the development of insulin resistance (Lee *et al*. 2010). It has also been reported that HOCl could induce phosphorylation of PKCζ, causing activation of NADPH oxidase in endothelial cells (Xu *et al*. 2006). Whether other PKC isoforms are involved in these processes requires additional investigation.

We have recently reported that exogenous HOCl treatment increased ONOO^−^ production in 3T3-L1 adipocytes and endothelial cells (Xu *et al*. 2006, Wang *et al*. 2014). ONOO^−^ plays a critical role in the pathogenesis of insulin resistance through multiple pathways. For instance, ONOO^−^ induces tyrosine nitration of insulin signaling proteins, including insulin receptor β and IRS1, leading to inactivation and degradation in adipocytes (Nomiyama *et al*. 2004). ONOO^−^ induces *S*-glutathionylation of p21ras and serine phosphorylation of IRS1 in endothelial cells as well (Clavreul *et al*. 2006). In this study, we describe a novel signal transduction mechanism by which HOCl-mediated insulin resistance is ONOO^−^ dependent. The ONOO^−^ scavenger uric acid offers considerable protection against HOCl-induced phosphorylation of PKCθ and IRS1-Ser307. Because ONOO^−^ is formed by the rapid reaction of NO with O_2_·^−^, O_2_·^−^ and NO inhibitors show similar protective effects on phosphorylation of inflammatory kinases. On the other hand, treatment with ONOO^−^ directly induces phosphorylation of PKCθ, leading to a reduction of tyrosine phosphorylation of IRS1 by insulin. These observations indicate that treatment with ONOO^−^ is essential for activation of inflammatory kinases, which triggers insulin resistance after stimulation with HOCl.

In conclusion, the current findings strongly indicate that HOCl is a novel contributor to the development of insulin resistance in adipocytes, and a clinically relevant concentration of HOCl induces production of ONOO^−^ and activation of inflammatory kinases, resulting in impairment of the insulin signaling pathway. HOCl-induced insulin resistance might represent a common pathological pathway in the development of the metabolic syndrome and type 2 diabetes.

## Author contribution statement

J Zhou and Q Wang contributed equally to the study design, performed experiments, and wrote the manuscript. Y Ding performed some experiments. M-H Zou contributed to the study design and interpretation and wrote the manuscript. M-H Zou is the guarantor of this work and, as such, had full access to all the data in the study and takes responsibility for the integrity of the data and the accuracy of the data analysis.

## Figures and Tables

**Figure 1:** HOCl induces insulin resistance in 3T3-L1 adipocytes. (A) HOCl dose dependently inhibits insulin-stimulated glucose uptake. Serum-starved 3T3-L1 adipocytes were pretreated with various concentrations of HOCl (0, 50, 100, 200, 500, and 1000 μmol/l) for 1 h and stimulated with 100 nmol/l insulin or left unstimulated for 15 min and then incubated with [^3^H]-2-deoxyglucose (2DG) for 5 min. Glucose uptake was evaluated from [^3^H]-2-DG counts in each cell lysate. Results are expressed as mean±s.e.m. (*n*=5, *P<0.05 and **P<0.01 vs no HOCl treatment). (B, C and D) HOCl impairs insulin signaling pathway. 3T3-L1 adipocytes were pretreated with 200 μmol/l HOCl for 1 h and stimulated with or without 100 nmol/l insulin for 15 min. Membrane proteins were isolated using the Mammalian Membrane Protein Extraction Kit (Abcam, Cambridge, MA, USA). Cell lysis was subjected to SDS–PAGE and immunoblotted with indicated antibodies (B and C). Cell lysates were immunoprecipitated using Akt antibody and immunoblotted with phospho-GSK3β for *in vitro* Akt kinase assay using non-radioactive Akt kinase assay kit (Cell Signaling Technology, Inc., Beverly, MA, USA) (D). The blot is a representative of results obtained from five independent experiments.

**Figure 2:** HOCl promotes phosphorylation of IRS1 at Ser307 in association with JNK and IKKα/β. 3T3-L1 adipocytes were pretreated with 200 μmol/l HOCl for 1 h before treatment with 100 nmol/l insulin for 15 min or being left untreated, and levels of expression of phospho-IRS1-Ser307 and phospho-IRS-Tyr612 (A), IKK (B), and JNK (C) were determined by western blot analysis. The blot is representative of results obtained from five independent experiments.

**Figure 3:** Inhibition of IKK blocks HOCl-induced serine phosphorylation of IRS1 and insulin resistance. (A) 3T3-L1 adipocytes were pretreated with 10 μmol/l PS1145 for 90 min and incubated with 200 μmol/l HOCl for 1 h and then stimulated with 100 nmol/l insulin or left unstimulated for 15 min. (B) 3T3-L1 adipocytes were transfected with IKKβ siRNA or control siRNA for 48 h and treated with 200 μmol/l HOCl for 1 h and then stimulated with or without 100 nmol/l insulin for 15 min. Western analysis of protein expression and phosphorylation of IKK, IRS1, Akt, and GSK3β was performed. Blots are representative of the results from five independent experiments.

**Figure 4:** Inhibition of JNK prevents HOCl-induced phosphorylation of IRS1 at Ser307 and insulin resistance. (A) 3T3-L1 adipocytes were pretreated with 30 μmol/l SP600125 for 90 min and incubated with 200 μmol/l HOCl for 1 h and then stimulated with 100 nmol/l insulin or left unstimulated for 15 min. (B) 3T3-L1 adipocytes were transfected with JNK2 siRNA or control siRNA for 48 h and treated with 200 μmol/l HOCl for 1 h, and then stimulated with 100 nmol/l insulin or left unstimulated for 15 min. Western analysis of protein expression and phosphorylation of JNK, IRS1, Akt, and GSK3β was performed. Blots are representative of the results from five independent experiments.

**Figure 5:** PKCθ mediates phosphorylation of IKK, JNK, and IRS1 and insulin resistance. 3T3-L1 adipocytes were transfected with PKCθ siRNA or control siRNA for 48 h and treated with 200 μmol/l HOCl for 1 h and subsequently stimulated with 100 nmol/l insulin for 15 min or left unstimulated. Western blot analysis of protein expression and phosphorylation of PKCθ, IKK, JNK, and IRS1 (A and B). Akt kinase activity in cell lysates was measured (C). The membrane fraction was isolated and proteins were subjected to SDS–PAGE and immunoblotted with GTLU4 antibody (D). The blots are representative of results obtained from five independent experiments.

**Figure 6:** HOCl mediates inflammatory kinase phosphorylation through ONOO^−^. (A and C) 3T3-L1 adipocytes were serum starved overnight, then treated with 200 μmol/l HOCl for 1 h in the presence of SOD1 (150 U/ml), l-NAME (1 mmol/l), or uric acid (UA, 50 μmol/l), followed by stimulation with 100 nmol/l insulin for 15 min. Cell extracts were immunoblotted with indicated antibodies. (B and D) 3T3-L1 adipocytes were serum starved overnight, then treated with ONOO^−^ (50, 100, and 200 μmol/l) for 1 h. Western blot analysis of protein expression and phosphorylation of PKCθ, IKK, JNK, and IRS1 was performed. The blot is a representative of blots obtained from five independent experiments.

**Figure 7:** HOCl-induced insulin resistance is ONOO^−^ dependent. 3T3-L1 adipocytes were serum starved overnight and treated with 200 μmol/l HOCl for 1 h in the presence of SOD1 (150 U/ml), catalase (100 U/ml), l-NAME (1 mmol/l), or uric acid (50 μmol/l), then stimulated with 100 nmol/l insulin for 15 min or left unstimulated. Cell extracts were immunoblotted with antibodies against IRS1 and Akt (A and B). Akt kinase activity in cell lysis was measured (C). Membrane proteins were isolated and then subjected to SDS–PAGE and immunoblotted with GTLU4 antibody (D). Blots are representative of results obtained from five independent experiments.

**Figure 8:** MPO deficiency prevents phosphorylation of IKK, JNK, and IRS1-Ser307 in WAT from HFD-fed mice. (A, C and D) WT and *Mpo* ^−^^*/*^^−^ mice were fed with ND or HFD for 16 weeks. Homogenates of epididymal WAT were prepared and levels of MPO, phosphorylation of IRS1, PKCθ, IKK, and JNK were analyzed by western blotting. (B) Expression of 3-chlorotyrosine in WAT was analyzed by using immunohistochemistry, magnification: 20×. (E) Schematic diagram of the relationship between for HOCl-induced phosphorylation of IRS at Ser307 and insulin resistance.

**Table 1:** Body weight and metabolic characteristics in WT mice and *Mpo* ^−^^*/*^^−^ mice after 16 weeks of HFD. Values are mean±s.e.m., *n*=7 for each group. Six-week-old male mice were fed a high-fat diet for 16 weeks. Blood was collected after 6 h of fasting and metabolic parameters were measured from serum.

	**WT**	***Mpo*^*−/−*^**
Initial body weight (g)	19.1±1.0	19.5±0.6
Final body weight (g)	44.5±4.2	40.1±2.8*
Fasting blood glucose (mmol/l)	10.5±1.1	7.8±0.8*
Fasting insulin (pmol/l)	258±25	134±18*
HOMA-IR (pmol/l×mmol/l)	5.4±0.1	2.7±0.1*
Food intake (mg/g body weight per day)	103±10	111±7

*P<0.05.
